# Analysis of Logistics Linkage by Digital Twins Technology and Lightweight Deep Learning

**DOI:** 10.1155/2022/6602545

**Published:** 2022-04-28

**Authors:** Liang Qiao, Ying Cheng

**Affiliations:** ^1^The Tourism College of Changchun University, Jilin Changchun 130607, China; ^2^Changchun SCI-TECH University, Jilin Changchun 130600, China

## Abstract

The present work expects to meet the personalized needs of the continuous development of various products and improve the joint operation of the intraenterprise Production and Distribution (P-D) process. Specifically, this paper studies the enterprise's P-D optimization. Firstly, the P-D linkage operation is analyzed under dynamic interference. Secondly, following a literature review on the difficulties and problems existing in the current P-D logistics linkage, the P-D logistics linkage-oriented decision-making information architecture is established based on Digital Twins. Digital Twins technology is mainly used to accurately map the P-D logistics linkage process's real-time data and dynamic virtual simulation. In addition, the information support foundation is constructed for P-D logistics linkage decision-making and collaborative operation. Thirdly, a Digital Twins-enabled P-D logistics linkage-oriented decision-making mechanism is designed and verified under the dynamic interference in the linkage process. Meanwhile, the lightweight deep learning algorithm is used to optimize the proposed P-D logistics linkage-oriented decision-making model, namely, the Collaborative Optimization (CO) method. Finally, the proposed P-D logistics linkage-oriented decision-making model is applied to a domestic Enterprise H. It is simulated by the Matlab platform using sensitivity analysis. The results show that the production, storage, distribution, punishment, and total costs of linkage operation are 24,943 RMB, 3,393 RMB, 2,167 RMB, 0 RMB, and 30,503 RMB, respectively. The results are 3.7% lower than the nonlinkage operation. The results of sensitivity analysis provide a high reference value for the scientific management of enterprises.

## 1. Introduction

Production and Distribution (P-D) are the two core links that directly affect the Enterprise (ENT)'s production efficiency and overall operation efficiency. Traditionally, P-D are operated independently by the production and logistics departments within an ENT or by the third-party logistics ENTs [1, 2]. P-D are two independent Decision-Making (DM) links with different objectives and constraints to maximize their respective interests. There is a lack of timely information sharing and operational coordination between the two links. In the traditional ENT DM process, a single link often ignores the actual situation of the other link, so it is not easy to optimize the overall operation [3, 4]. Therefore, global optimization and joint operation of P-D are essential to maximize operational efficiency and operation cost and maintain high-level customer service for ENTs [5].

In recent years, P-D-oriented Collaborative Optimization (CO) from a global perspective has attracted the extensive attention of scholars and production ENTs. Scholars study the optimization of P-D parameters under different customer demand and delivery parameters. Loro et al. [6] used activity-based cost to study the collaborative logistics process and its implementation in electronics and household appliances and evaluated the benefits. They associated each activity with its appropriate cost driver and implemented the analytical simulation model. Guo et al. [7] proposed a Self-adaptive Collaborative Control (SCC) mode to enhance the intelligence, flexibility, and elasticity of the intelligent production logistics system. They collected and processed data using Cyber-Physical Systems (CPS) and Industrial Internet of things (IIoT) to implement DM and optimization. They also simulated the dynamic behavior of physical manufacturing resources (such as machines and vehicles in the workshop) by hybrid automata to overcome the shortcomings of the CO algorithm. The results showed that the proposed method shortened the waiting and completion time and reduced Energy Consumption (EC). Zhao et al. [8] analyzed the multiobjective scheduling in logistics distribution and implemented a multiobjective bilevel programming model. In addition, they used the genetic strategy of genetic factors for rapid advantage ranking. They figured out an optimal path for distributing vehicles, providing a reference for optimizing the logistics distribution path.

Based on the above research, in Intelligent Manufacturing (IM), the integrated optimization method is mainly used to optimize P-D. Therefore, combined with the actual production distribution operation problem, this paper expands the application of the Digital Twins from independent objects to multiple related objects' optimization. It makes up for the lack of research on global correlation twinning in complex multiunit production and operation systems in the past. It enriches the application scenario of Digital Twins.

## 2. Related Works

### 2.1. Digital Twins

The intelligent enabling technologies provide a solid basis for online collaboration and independent DM of P-D. Digital Twins technology features excellent characteristics, such as data-driven process, iterative optimization, real-virtual integration, and real-time interaction. These features also meet the needs of the current research problems. Thus, this paper intends to use Digital Twins intelligent technology to support the linkage Production-Distribution (PD) DM.

Digital Twins was first proposed by professor Grieves of the University of Michigan in 2003. At that time, Grieves defined Digital Twins as a Three-Dimensional (3D) model including virtual products, physical products, and their connection. Over time, scholars continue to supplement and improve the connotation of Digital Twins. For example, the National Aeronautics and Space Administration (NASA) claims Digital Twins to be a highly integrated simulation model for aerospace vehicles. Digital Twins can map or reflect the real-time operation state, future evolution trend, and basic functions of entity objects in the computer information world. It usually employs historical data, real-time sensing data, and physical models.

Based on the Digital Twins, foreign scholars have designed a Manufacturing Execution System (MES) to integrate data from two different sources: machine tool operation data and production execution data. The MES realizes data-driven production optimization. Noticeably, Digital Twins technology can also combine knowledge learning technology to improve reasoning ability by extracting and reasoning relevant knowledge from production data. As a result, the Digital Twins system can improve the manufacturing process and production management.

Arguably, Digital Twins technology provides a feasible technical framework and management mode for the interactive control and digital construction of physical entities. Digital Twins technology is mainly used to optimize and control a single independent object. However, there is still a lack of research on online collaborative decision control and global correlation virtual twins for multiple correlated physical objects.

### 2.2. Multidisciplinary Design Optimization Method

Under the customized production model, the demand uncertainty can lead to a significant increase in the complexity of P-D joint operation. At the same time, all links in the P-D process tend to make independent decisions. The traditional integrated optimization method is challenging to solve the P-D collaborative problem under dynamic interference. Therefore, a distributed DM-oriented CO approach must be devised for ENT P-D.

MDO, proposed in 1982, is an effective global optimization methodology for designing and optimizing complex systems by analyzing the synergy and interaction between large-scale complex systems and their multiple subsystems. Over the years, the MDO method has been widely used in the design and optimization of large and complex equipment, such as automobile, aerospace, and machinery, as well as Supply Chain (SC) operation. According to the decomposition levels, complex systems are divided into single-level MDO, two-level MDO, and multilevel MDO. Single-level MDO mainly includes All At Once (AAO) and feasible multidisciplinary methods. By comparison, two-level MDO methods (such as CO method) and multilevel MDO methods include the target cascade method and Lagrange coordination. P-D linkage operation can be decomposed into a two-level coordination optimization problem, so the present work focuses on the research progress of CO methods.

The CO method decomposes the complex system optimization into a two-level optimization problem of system-level and multiple-discipline levels. Under the coordination of system-level, discipline level can realize distributed parallel optimization. The CO method has the characteristics of high efficiency, rapidity, simplicity, and organization form of design division in line with the actual project. It has become one of the more studied MDO methods. Like most methods, the CO method includes theoretical and applied research.

Theoretically, scholars have studied how to improve the solution performance and practicability of the CO method. The CO method can be optimized either by equality constraint relaxation or the Response Surface Method (RSM). These improvements effectively improve the solution efficiency of the CO method. The application and research of the CO method in large-scale system optimization mainly stay in the static design optimization of collaborative structure and parameters. There is less research on CO method-based dynamic modeling and online DM for the complex multiunit system.

### 2.3. Collaborative Optimization of P-D

CO of P-D refers to comprehensively considering the actual production, inventory, and distribution situation, formulating the optimal P-D cooperation plan, meeting customer needs with the minimum total operation cost, and improving market competitiveness. The P-D-oriented CO includes production scheduling and distribution allocating. Production scheduling is responsible for formulating the order production sequence, determining the start processing time, and allocating production resources. By contrast, distribution allocation determines the distribution start time of Finished Products (FPs) and formulates the distribution sequence for each order. It then administers vehicles to undertake distribution tasks and plans distribution routes. The overall operation cost of SC can be effectively reduced by coordinating production scheduling and distribution allocation.

The existing research on P-D-oriented CO is mainly carried out in a stable production and operation environment. There is less research on P-D's dynamic, collaborative operation under the uncertain production and operation environment. In addition, P-D mainly uses the integrated optimization method. The study is still very few on the P-D-oriented multiunit distributed CO method under the dynamic operational environment.

### 2.4. Analysis of the Logistics Linkage System

Here, the logistics linkage system is optimized based on Digital Twins and optimization algorithms [9, 10]. Based on the traditional digital modeling and simulation technology and thanks to the advancement of Information Technology (IT), Digital Twins technology can effectively solve some problems in the operation process of production ENTs. The integrated Digital Twins technology has the following three characteristics. (1) Digital Twins can obtain the personnel, equipment, and materials in the whole P-D operation and environmental data. They can also integrate and obtain various real-time data of physical entities, which is an accurate image of physical entities. (2) Digital Twins can accurately describe the physical entity and optimize the physical entity based on the optimization model. It makes up for the deficiency that the traditional modeling and simulation methods only pay attention to accurately reflecting the physical object's basic characteristics and running state. (3) Digital Twins technology realizes real-time physical-digital interaction through the whole Life Cycle (LC) of physical entities. It also realizes the coevolution of digital objects and physical entities through the continuous accumulation of relevant knowledge. Technically, Digital Twins can improve themselves with no limit. The unique advantages of Digital Twins enable it to collect data from multiple dimensions such as personnel, equipment, materials, process, and environment. Thus, Digital Twins can accurately present the real operation state of physical objects in the computer-based information world. Meanwhile, they can conduct virtual simulations driven by real-time data to generate the optimal linkage operation strategy and realize the dynamic control of P-D. Thereupon, this paper uses Digital Twins technology to support the P-D linkage-oriented DM under dynamic interference and constructs the Digital Twins-enabled P-D linkage-oriented DM information architecture.

Logistics linkage is a process including P-D links, with each link affecting one another and the overall system stability. Therefore, the collaborative process and high relevance of all logistics links are the basis for ensuring the efficiency of the P-D links [11, 12]. In particular, a dynamic environment-robust P-D logistics linkage can improve the logistics system's anti-interference ability and efficiency [13].

### 2.5. The Basic Process of P-D Logistics Linkage

P-D logistics linkage involves an interrelated but self-sustained set of dynamic production, storage, and distribution link. Remarkably, the production link manufactures customization products (home-deliverable over the distribution link). It involves multiple departments [14, 15], among which the workshop is a decision maker. Differently, the logistics company makes decisions in the distribution link [16]. The structure of the P-D logistics linkage is shown in Figure 1.

As in Figure 1, the P-D logistics linkage operation process is described below. (1) Multiple customers submit orders according to product sales to the customer service department. The demand order information generally includes customer name, product type, product quantity, delivery date, and more. The customer service department integrates the demand orders received from multiple customers, formulates production orders and shipping orders, releases the production orders to each production workshop and warehouse, and releases the shipping orders to the third-party logistics company [17]. (2) According to the production orders issued by the customer service department, multiple production workshops fabricate different types of products by arranging the production time, production sequence, production quantity, and production equipment. (3) Due to the extremely limited buffer space at the offline point of the production workshop, the forklift can transport the FPs to the FPs' warehouse in time to avoid affecting the continuity of production. (4) The warehouse allocates the storage space according to the production order issued by the customer service department. Then, it uses the stock arrangement rules to meet the storage requirements of offline FPs. In the actual implementation, the FPs are stored on the pre-allocated cargo way through the forklift in the factory. Finally, checkout and delivery are arranged after all the FPs of the same customer order are ready [18]. (5) The third-party logistics company formulates the distribution plan according to the delivery note issued by the customer service department and arranges the distribution vehicles according to the loading principle. Then, it loads and departs the FPs in the warehouse and starts the distribution of FPs according to the optimal distribution route after all the FPs are loaded [19].

### 2.6. Operation of P-D Logistics Linkage

The P-D logistics linkage is subject to the P-D departments' decisions. For example, a short supply of raw materials will cause production suspension, thus extending the product output time. The distribution vehicle failure or traffic jams can also hinder products' on-time delivery. Insufficient cooperation of P-D links might cause associated overstock and broken FP inventory, which adds up the overall production and operation costs. The random dynamic interference generated in production execution harms the P-D operation [20, 21]. The main problems include the following:

- Uncertain production completion time. The complex production and operation process includes various production factors, such as personnel, materials, equipment, and technology. The change of each production factor may affect regular production and operation. Significant uncertainty makes the production operation vulnerable to dynamic interference, thus significantly increasing possible mismatch in production factors and affecting the normal operation. As a result, it prevents the accurate control of the product production process, resulting in large fluctuations in the offline time and offline quantity of products.
- Long queueing time for order completion. Personalized demand orders often contain multiple types of products. Due to the universal application of professional division of labor in production ENTs, customers' orders are usually re-distributed into different production workshops. They can be delivered until all production workshops complete the products order and the warehouse is ready. However, due to random dynamic interference, the offline time of products in each production workshop fluctuates significantly. Thus, each production workshop's offline time cannot be synchronized, resulting in a long queueing time in the warehouse, increasing the storage cost.
- The operation efficiency of FP distribution is low. The number of distribution vehicles owned by third-party logistics companies is extremely limited. When the uncertainty of offline order production is more significant, the demand for distribution vehicles will be more unpredictable. Given the random uncertainty, it is difficult for the third-party logistics company to effectively integrate the distribution demand of each order to realize the scale effect. In that case, low vehicle loading rate and long distribution path occur from time to time. At the same time, due to the great uncertainty of products offline, the offline FPs have no vehicles to match sometimes. It is necessary to pay a huge penalty fee for delayed delivery, which will affect customer satisfaction in the long run.
- Poor execution of production plan and distribution plan. The randomness and dynamics often lead to dynamic changes in P-D's execution and operation environment. Under such circumstances, the production scheduling plan and FP distribution plan are challenging to meet the operation requirements of the actual site. At the same time, due to the lack of real-time and effective coordination and response mechanisms and methods among the DM links of P-D, the implementation effect of the initial plan is poor.

### 2.7. Architecture and Mechanism of the P-D Logistics Linkage DM Based on DT

#### 2.7.1. Architecture of P-D Linkage DM under Digital Twins

P-D logistics linkage operation is a complex process including multiple independent DM units. The highly efficient operation is inseparable from each object-specified and constrained DM unit [22, 23]. Usually, a single DM link fails to consider the actual operation of other related links, so the relevant decisions can only achieve its local optimization.

The production link's main DM goal is to consider the actual personnel, materials, equipment, and other resources in the production workshop. DM can help formulate the production scheduling plan with optimal resource allocation and complete the production requirements of customer orders. In making the production scheduling plan, it is unclear whether the resources and capabilities of the storage link and distribution link can meet the planning requirements.

The main DM goal of the storage link is to maximize the utilization rate of storage space and warehouse turnover to complete the storage of FPs. It does not consider whether its operation scheme benefits the production and distribution links.

For the distribution link, the main DM goal is to distribute the FPs from the warehouse to each customer with the maximum vehicle loading rate, the minimum distribution cost, or the shortest distribution path according to the existing vehicle resources (model and number of vehicles). Generally, the actual situation of production and warehouse operations is not considered, resulting in the inability to optimize time or cost from the system's perspective.

Digital Twins-enabled P-D linkage-oriented DM can accurately describe physical entities and reflect their essential characteristics [24, 25], as depicted in Figure 2.

As in Figure 2, the Digital Twins-enabled P-D linkage DM architecture is divided into physical object layer, virtual object layer, linkage service layer, and linkage application layer from top to bottom. The four levels are described as follows:

The physical object layer uses Intelligent Sensing Technologies (IST), such as Radio Frequency Identification (RFID) tag, RFID reader, Global Positioning System (GPS) device, and Personal Digital Assistant (PDA) handheld device to sense the multidimensional real-time operation data of personnel, equipment, materials, process, and environment generated in the P-D process in real time. It also provides data support for each DM unit's interconnection, cooperative operation, and linkage DM.

The virtual object layer supports online linkage DM through an accurate virtual image of physical objects and dynamic virtual simulation of digital objects. The virtual image maps the whole production process based on the geometric and relational models. It is reconstructed using the multidimensional and real-time production operation data to present the actual operation of physical objects in the information world. Virtual simulation makes accurate and comprehensive operation effect judgment on the production system according to the real-time image data and constantly iterates and optimizes the linkage DM strategy to support the online linkage DM.

The linkage service layer is driven by virtual simulation data and independently analyzes and discriminates the execution process of P-D and the behavior of resources. Meanwhile, it provides intelligent production scheduling DM service and intelligent vehicle scheduling DM service. Thus, the adaptive DM is realized to control the whole P-D process.

The linkage application layer provides a Human-Computer Interaction (HCI) application system with complex production and operation systems and multiunit joint operations. Users interact with the application system through the intelligent mobile terminal or Personal Computer (PC) to make online linkage decisions to reduce the adverse impact of dynamics on the production system.

In summary, P-D logistics linkage mainly involves three objects: production workshop, warehouse, and distribution vehicle.  Figure 3 specifies the three objects' relevant equipment's operating environment.

As in Figure 3, the three objects include the business process, digital environment, the sensing device, and physical environment.

Production workshop is the core component of P-D operation. The real-time acquisition of its dynamic data directly affects the efficient linkage between P-D. Production workshops can install intelligent sensing devices on production equipment and pastes RFID tags on material and FP pallets. It can equip workshop operators with intelligent wearable devices and install RFID readers at stations and workshop offline points. Besides, it can provide Wireless Sensor Networks (WSNs), such as Fourth Generation (4G)/Fifth Generation (5G) networks and WiFi. Thus, the workshop data can be accurately obtained and transmitted in real time, including personnel, materials, and environment.

The FP warehouse is the buffer in the P-D operation process, which determines the continuity and smoothness of P-D. The FP warehouse can place a mobile access control system at the door like the production workshop. Meanwhile, the workshop can paste bar codes on the shelves and equip forklift drivers with onboard tablet computers. It can also configure readers for warehouse staff and cover antennas, 4G/5G, and other wireless transmission networks in the whole warehouse. As such, real-time operation data can be obtained, including the use of cargo spaces, the FP storage information, and the access of forklifts in and out.

*(1) Distribution Vehicle*. The relevant parameter data and dynamic operation data of distribution vehicles are an essential basis for the linkage operation of P-D. Specifically, tablet computers can obtain real-time cargo loading and unloading data and customer location. The dynamic operation data, such as the position, speed, and loading rate of distribution vehicles, are obtained in real-time through GPS technology.

#### 2.7.2. Digital Twins-Enabled P-D Linkage DM Mechanism

Supported by P-D linkage DM architecture, a P-D logistics linkage DM mechanism is proposed, as in Figure 4.

The Digital Twin-enabled P-D linkage-oriented DM mechanism is divided into three main linkage stages: initial planning stage, dynamic revision planning stage, and dynamic coordination and control stage. The specific description is as follows:

  Initial planning stage. Before production, IST can collect and integrate real-time operation data, such as personnel, equipment, materials, methods, and environment, in the whole P-D process. Driven by real-time fusion data, the virtual object layer in the multiunit linkage DM architecture based on Digital Twins simulates the linkage DM model. The model aims to achieve the minimum total system cost. It plans the optimal collaborative initial work through the linkage DM of multiple independent DM units with heterogeneous DM structures and control objectives.
  Dynamic revision planning stage. In P-D, the virtual object layer in the Digital Twins-enabled linkage DM architecture accurately reflects the production and operation environment. Then, it dynamically simulates, evaluates, and optimizes the whole process based on relevant models. At the same time, the execution deviation is obtained by comparing the actual operation state of the system with the dynamic optimization state. According to the deviation value, four online linkage decisions are triggered: internal rescheduling linkage of the unit, rescheduling linkage of the associated unit, system resource reconfiguration linkage, and customer demand readjustment linkage. These online linkage decisions maintain the performance of the P-D system in the feasible optimal state under dynamic interference.
  Dynamic coordination and control stage. Feeding back the linkage DM results of dynamic revision planning to relevant units in real time realizes the real-time online adjustment of the production system. The whole process of production execution is a timely, adaptive, and feasible optimal state of system control under the dynamic action.

Based on the real-time perception of the dynamics of the production execution environment, the linkage control scheme is continuously revised and optimized to eliminate the adverse interference of the dynamics to the production system and realize the coordinated management and control of the whole KC of the complex production system.

### 2.8. Optimization Methods

The methods of implementing the P-D logistics linkage mathematical model are introduced. The two-level CO is used for systematic coordination in distributed DM and global optimization to avoid the active interference of P-D linkage information.

#### 2.8.1. Introduction to CO

Collaborative Optimization (CO) is a two-level optimization method that can effectively solve the coupling problem of large-scale complex systems. It decomposes the complex optimization design problem into a two-level structure, a multiple parallel discipline level and a system level. It can solve the coupling problem between different disciplines by simplifying their relationship. Due to its high efficiency, rapidity, simplicity, and many other characteristics, CO has been successfully applied in many fields, such as aerospace equipment manufacturing, automobile manufacturing, mechanical equipment design, and supply chain optimization [26, 27].

#### 2.8.2. Genetic Algorithm (GA)

American scholars proposed GA in the early 1970s, inspired by the theory of evolution. GA has many advantages, such as simple principle, easy operation, strong universality, and robust global optimization ability. It is widely used in solving and optimizing large-scale complex combinatorial optimization problems [28, 29]. The composition of GA is unfolded in Figure 5:

As in Figure 5, GA is composed of six elements. Among them, individual coding converts the problem to be solved into genetic space according to the relevant principle. Its coding methods include binary coding (0 and 1), real-number coding, and symbolic coding. The operation steps of GA are presented in Figure 6 [30, 31].

GA can solve practical problems by simulating biological evolutionary processes in nature. It determines the optimal solution to practical problems through repetitive genetic operations and refers to some biogenetics knowledge and terms. In biogenetics, biological evolution is realized through the continuous crossover and mutation of chromosomes in biological individuals. The chromosomes in GA have two expression forms: genotype and phenotype. Genotype refers to the various gene strings making up individual chromosomes, and phenotype is the form in vitro of organisms made up of chromosomes. Fitness (adaptability) is borrowed from the biological concept of individuals adapting to their living environment. According to Darwin's Survival of the Fittest (SOTF) theory, only biological individuals with stronger adaptability can survive. Then, they inherit and evolve through gene mutation and recombination. When GA is used, feasible solutions to practical problems are called chromosomes, and genes are elements of chromosome coding, which mainly represent the characteristics of individuals. GA cannot directly solve practical problems through genetic operations. Therefore, to use GA to solve practical problems, it is necessary to convert the problem parameters into the chromosomes in the GA. This conversion process is called coding. On the contrary, converting the GA individuals into the actual problem solutions is called decoding.

Compared with the traditional optimization algorithm, GA has the following characteristics:

1. Broader search scope: Traditional optimization algorithms usually calculate a single initial value when solving practical problems. Thus, it has a slow operation and cumbersome solution process. In contrast, GA solves problems in a larger domain through population search. As a result, the problem becomes easier to solve, and GA can calculate quickly with high precision.
2. Probabilistic search over deterministic search: GA uses a certain probability to search the individual population and randomly search for the optimal solution of the problem. Such a mechanism improves optimization efficiency. Conversely, the deterministic search method easily misses individuals with high fitness, thus missing the optimal solution.
3. Fitness-based search: When solving practical problems, GA first constructs the fitness function and determines the search range and direction accordingly to fitness. There is no need to determine the search direction through Objective Function (OF)'s derivation, so the search efficiency is greatly improved.
4. Strong expansibility: GA can combine with other optimization algorithms to complement one another, give full play to their advantages, and improve the ability and efficiency of solving optimization problems.

In nature, biological individuals follow the natural law of SOTF. Biological individuals with strong adaptability have a high probability of survival against a dynamic natural environment. Therefore, these individuals can inherit excellent genes and pass them down to the next generation. GA is established based on biological evolution theory. Similarly, in GA-based optimization problems, the fitness represents the quality of the problem solution. The greater the fitness is, the better the gene individual is, and the closer it is to the optimal solution. The fitness is calculated through the fitness function. Thus, fitness function design has a certain impact on GA's operation efficiency and solution accuracy. Therefore, it is necessary to design an appropriate fitness function. Generally, there are the following methods to design a fitness function:

(1) Direct conversion
Fitness function can be directly converted from OF, thus the direct conversion method. Equation (1) gives the solution of the OF maximization problem:
  (1) $$\begin{array}{c} F_{\left(x\right)}=f_{\left(x\right)}. \end{array}$$
Likewise, equation (2) gives the solution of the OF minimization problem:
  (2) $$\begin{array}{c} F_{\left(x\right)}=-f_{\left(x\right)}. \end{array}$$
The direct conversion method is relatively simple and convenient to operate, but there are some shortcomings. For example, the direct conversion uses the roulette selection that demands a nonnegative function value. Still, the fitness cannot always be calculated as nonnegative.
(2) Boundary construction
The boundary construction is an improved direct conversion method. It designs the fitness function by adding the corresponding boundary value, divided into two cases.
Equation (3) gives the solution of the OF maximization problem:
  (3) $$\begin{array}{c} F_{\left(x\right)}=\left\{\begin{array}{cc} f_{\left(x\right)}-C_{\text{min}}, & f_{\left(x\right)}\geq C_{\text{min}},\\ x, & \text{other.} \end{array}\right. \end{array}$$
Equation (4) gives the solution of OF minimization problem:
  (4) $$\begin{array}{c} F_{\left(x\right)}=\left\{\begin{array}{cc} C_{\text{max}}-f_{\left(x\right)}, & C_{max}\geq f_{\left(x\right)},\\ 0, & \text{other.} \end{array}\right. \end{array}$$
In equation (4), *C*_min_—OF minimum estimation; *C*_max_—OF maximum estimation.

## 3. Implementation of the P-D Logistics Linkage DM Model

### 3.1. P-D Logistics Linkage Model Based on CO

This section discusses the optimization modeling of P-D links. The optimization of the P-D linkage model is as follows. (1) A low-cost plan is formulated according to customers' requests. (2) Then, the dynamic process is modified in the P-D link, reducing the cost of the whole system. After that, the following hypotheses are put forward, as listed in Tables 1 and 2.

As mentioned above, the CO-based P-D logistics linkage system aims to reduce the target difference between the P-D subsystem and minimize the whole system's cost. The cost is reduced by:

(5) $$\begin{array}{c} \min f\left(Z\right)=Z_{p}^{2}+Z_{dt}^{2}. \end{array}$$

The OF is counted by equation (5) to minimize the operation cost of the whole system.

(6) $$\begin{array}{c} J_{p}^{*}={\left(Z_{p}-Z_{p}^{*}\right)}^{2}\leq \varepsilon , \end{array}$$

(7) $$\begin{array}{c} J_{d}^{*}={\left(Z_{dt}-Z_{d}^{*}\right)}^{2}\leq \varepsilon , \end{array}$$

(8) $$\begin{array}{c} Z_{p}^{*}=\sum_{p=1}^{P}\left[{\text{FC}}_{\text{pro}}^{p}+\sum_{i=1}^{n}\sum_{j=2}^{\prime }\left(t_{e_{ij}}^{p}-t_{e_{ij-1}}^{p}\right){\text{VC}}_{\text{pro}}^{p}\right], \end{array}$$

(9) $$\begin{array}{c} z_{\dot{d}}^{*}=\overset{m}{\underset{k=1}{\sum }}FC_{dis}^{k}+\overset{m}{\underset{k=1}{\sum }}\overset{c}{\underset{a=1}{\sum }}\overset{c}{\underset{b=1}{\sum }}y_{abk}d_{ab}{\text{VC}}_{\text{dis}}^{k}+\lambda \left[\overset{c}{\underset{c=1}{\sum }}\max\left({\text{ET}}_{c}-T_{c},0\right)+\overset{c}{\underset{c=1}{\sum }}\max\left(T_{c}-{\text{LT}}_{c},0\right)\right]+\overset{P}{\underset{p=1}{\sum }}\overset{n}{\underset{i=1}{\sum }}{\text{VC}}_{\text{war}}Q_{i}^{p}t_{\text{war,}}^{p}. \end{array}$$

Equations (6) and (7) calculate system consistency constraints, equation (8) counts the production cost of the subsystem, and equation (9) is for the distribution cost of the distribution system. In equation (9), ∑_*k*=1_^*m*^FC_dis_^*k*^ is the fixed vehicle allocation cost, ∑_*k*=1_^*m*^∑_*a*=1_^*c*^∑_*b*=1_^*c*^*y*_*abk*_*d*_*ab*_VC_dis_^*k*^ is the variable vehicle allocation cost, ∑_*p*=1_^*P*^∑_*i*=1_^*n*^VC_war_*Q*_*i*_^*p*^*t*_war,_^*p*^ is the inventory cost, and [∑_*c*=1_^*c*^max(ET_*c*_ − *T*_*c*_, 0)+∑_*c*=1_^*c*^max(*T*_*c*_ − LT_*c*_, 0)] is the distribution liquidated damages.

According to the above hypotheses, the production subsystem model is optimized, and the subsystem optimization mathematical model is implemented by:

(10) $$\begin{array}{c} \min:\max\left(t_{\text{off},i}^{p}|i=1,2,\ldots ,n+\alpha_{T}\right). \end{array}$$

Equation (10) is used to count the OF, so that the subsystem can be optimized and the production time can be the minimum.

Then, the distribution subsystem model is optimized by:

(11) $$\begin{array}{c} \min:\overset{m}{\underset{k=1}{\sum }}{\text{FC}}_{\text{dis}}^{k}+\overset{m}{\underset{k=1}{\sum }}\overset{c}{\underset{a=1}{\sum }}\overset{c}{\underset{b=1}{\sum }}y_{abk}d_{ab}{\text{VC}}_{\text{dis}}^{k}+\lambda \left[\overset{c}{\underset{c=1}{\sum }}\max\left({\text{ET}}_{c}-T_{c},0\right)+\overset{c}{\underset{c=1}{\sum }}\max\left(T_{c}-{\text{LT}}_{c},0\right)\right]+\overset{p}{\underset{p=1}{\sum }}\overset{n}{\underset{i=1}{\sum }}{\text{VC}}_{\text{war }}Q_{i}^{p}t_{\text{war},i}^{p}. \end{array}$$

Equation (11) is the optimization OF of the distribution subsystem, which is used to count the minimum costs, and the constraints are established by:

Distribution vehicle capacity constraints are calculated by:

(12) $$\begin{array}{c} \sum_{c=1}^{c}z_{ck}Q_{c}\leq Q_{k},\forall k\in K. \end{array}$$

Vehicle uniqueness constraints are calculated by:

(13) $$\begin{array}{c} \overset{m}{\underset{k=1}{\sum }}z_{ck}=1,\forall c\in V,c\neq 0,\\ \overset{c}{\underset{a=0}{\sum }}y_{abk}=z_{bk},\forall b\in V,\forall k\in K,b\neq 0,\\ \overset{c}{\underset{b=1}{\sum }}y_{abk}=z_{ak},\forall a\in V,\forall k\in K,a\neq 0. \end{array}$$

Constraints on vehicles returning to warehouse after delivery are calculated by:

(14) $$\begin{array}{c} \overset{C}{\underset{a=1}{\sum }}y_{aak}=1,\forall k\in K,\\ \overset{C}{\underset{a=1}{\sum }}y_{a0k}=1,\forall k\in K. \end{array}$$

Vehicle consistency constraint:

(15) $$\begin{array}{c} \sum_{a=0}^{C}y_{ack}=\overset{c}{\underset{b=1}{\sum }}y_{cbk},\;\forall c\in V,\;k\in K,\;c\neq 0. \end{array}$$

Vehicle delivery time constraints:

(16) $$\begin{array}{c} y_{abk}\left(T_{a}+s_{a}+t_{ab}-T_{b}\right)\leq 0,\;\forall k\in K. \end{array}$$

Order delivery constraints:

(17) $$\begin{array}{c} \max\left(t_{in,i}^{p}|p=1,2,\ldots ,P\right)\leq t_{\text{out },i}^{p},i=1,2,\ldots ,n+\alpha_{T}. \end{array}$$

### 3.2. P-D Logistics Linkage Model Based on GA

According to the research problem, the production subsystem and distribution subsystem models are simulated and solved by GA.

(1) Coding
The coding rule is: if there are three orders to be processed, each order has three processes, each process has 2, 2, and 3 parallel processing machines, and the numbers are 1, 2, 1, 2, 1, 2, and 3, respectively, a real-numbered double-layer matrix is generated:
  (18) $$\begin{array}{c} \left[\begin{array}{c} 231231321\\ 132231212 \end{array}\right]. \end{array}$$
In matrix equation (18), the first line is the operation of order 2, and the second is the third operation of order 3.
(2) Initializing population
Determine the chromosome length as ∑_*i*=1_^*n*^*Q*_*i*_, and the population size is between 50 and 500, forming the initial population.
(3) Fitness function
Here, the OF of minimizing the related costs of the distribution subsystem is taken as the fitness function.
  (19) $$\begin{array}{c} f=\overset{m}{\underset{k=1}{\sum }}{\text{FC}}_{\text{dis}}^{k}+\overset{m}{\underset{k=1}{\sum }}\overset{r}{\underset{a=1}{\sum }}\overset{r}{\underset{b=1}{\sum }}y_{abk}d_{ab}{\text{VC}}_{\text{dis}}^{k}+\lambda \left[\overset{c}{\underset{c=1}{\sum }}\max\left({\text{ET}}_{c}-T_{c},0\right)+\overset{c}{\underset{c=1}{\sum }}\max\left(T_{c}-{\text{LT}}_{c},0\right)\right]+\overset{p}{\underset{p=1}{\sum }}\overset{n}{\underset{i=1}{\sum }}vc_{\text{war}}Q_{i}^{p}t_{\text{war},i}^{p}. \end{array}$$
(4) Genetic evolutionary operation
  (a) Cross operation
  Two-point crossover is used to cross chromosomes, as shown in Figure 7.
  Crossover operation is the main way to maintain population diversity, effectively solving premature convergence. The steps are as follows. Based on the set crossover probability, select a crossover mode in line with the characteristics of the problem, and exchange some loci of the paired parent individuals selected by the selection operation. The basic GA usually adopts single-point crossover or multipoint crossover. Neither of these operations can guarantee the legitimacy of the second layer machine code.
  (b) Mutation operation
  In the first layer, two-point reciprocity is used for chromosome mutation, as illuminated in Figure 8.
  The specific steps of mutation operation are as follows: the first step is to randomly select a crossed chromosome and randomly select a mutant gene on the chromosome machine code. Then, the second step randomly generates a random number, compares the generated random number with the crossover probability, and decides whether to carry out a mutation operation. Suppose the random number is less than the mutation probability. In that case, the mutation is selected. A machine number is randomly selected from the remaining available parallel processing machine set according to the process number corresponding to the gene. Finally, the machine number chosen is replaced with the mutated gene.
(5) Optimization of constraint rules
The mathematical model of the distribution subsystem is solved on the maximum iteration, and the optimization results are output.

### 3.3. Optimization of P-D Logistics Linkage

Figure 9 describes the CO of the P-D logistics linkage system.

As in Figure 9, CO is divided into four steps: (1) Determining the initial design variable *Z*^*∗*^ and transferring it to the distribution and production subsystem; (2) Conducting internal optimization to obtain optimal solutions *Z*^*∗*^_*p*_ and *Z*^*∗*^_*d*_; (3) Getting optimal solution *Z′* of the system according to the optimal solution; and (4) Judging whether optimal solution Z′ conforms to penalty factor *ε*. If not, the iteration continues until the system consistency constraint is met.

## 4. Case Analysis of P-D Logistics Linkage Strategy

### 4.1. Case Result Analysis

This section employs the proposed P-D logistics linkage optimization model to a large domestic coating ENT H. Then, a case study is conducted using the Matlab simulation platform and comparative analysis. ENT H is a well-known coating manufacturer in China. Since its establishment, it has been deeply engaged in the Research and Development (R&D), production, and sales of coating products for a long time. Due to the large variety of coating products and its seasonal market demand, the demand for different coatings will fluctuate greatly. Then, to avoid the operation risk from market fluctuation, H ENT adopts the Make-To-Order (MTO) production mode. MTO can reduce the inventory of products while meeting customer needs.

Due to the gaps in coating products' physical and chemical properties, coating products have different requirements for production equipment and the environment. According to the characteristics of coating products, coating ENTs choose to arrange various kinds of products in other production workshops. At present, ENT H has three production workshops capable of producing three types of coating products: exterior wall paint, interior wall paint, and wood paint. After accepting the customers' orders, the customer service department will split the orders per product type and release the production requirements of different products to the corresponding production workshops. Then, the FPs will be transported by the forklift to the FP warehouse for temporary storage until all products in the same customer's order are ready. The third-party logistics company will arrange the distribution vehicles to distribute the FPs to the customers.

ENT H adopts the MTO production mode. Such a model can respond to customer needs to a certain extent. Yet, as people's life pursuit sublimes and vision broadens, more people choose personalized coating products over traditional mass production products. Generally, personalized demand features small-batch, multiple varieties, high timeliness requirements, and high randomness. Thus, it makes the production and operation of ENT H vulnerable to dynamic interference from orders, resources, and quality. This condition challenges ENT H's operations and unveils its low production efficiency, distribution, operation plan, and high production and operation cost. So far, almost all ENTs face dynamic customer demands during production execution, which dramatically affect the efficient implementation of production operation of ENT H. The dynamic customer demands faced by ENT H mainly include the following three situations:

(1) Temporary order increase. Simply put, customers add a new order based on the original demand order. (2) The demand quantity of the original order increases. That is, the order that has been planned or is being produced dynamically increases in quantity. (3) The demand quantity of the original order decreases. In other words, the order quantity reduces for the products being planned or produced. The first case has the most significant impact on the P-D operation in the MTO mode, and the probability of occurrence is greater than the latter two. Therefore, this paper studies the P-D linkage operation of ENT H under the interference of dynamic new demands to prove the effectiveness of the proposed linkage DC method.  Table 3 tabulates some information about the case.

Basic information of customers is plotted in Figure 10.

The basic information of distribution vehicles is manifested in Figure 11.

The optimization results of vehicle scheduling initialization are charted in Figure 12. Path number A: [0–9 (10) - 2 (14) - 13 (14) - 0], path number B: [0-1 (11) - 8 (11) - 15 (13) - 14 (13) - 0], path number C: [0–4 (12) - 11 (13) - 6 (14) - 10 (18) - 0], and path number D: [0–7 (17) - 12 (15) - 5 (16) - 3 (14) - 0].

As in Figure 12, an 8T vehicle distributes three orders 9, 2, and 13, and its load rate is 95%. A 10T vehicle distributes four orders 1, 8, 15, and 14, with a load rate of 96%. A 13T vehicle distributes four orders 4, 11, 6, and 10, with a load rate of 88%. Another 10T vehicle distributes three orders 7, 12, and 3, and its load rate is 95%. The average load rate of the four distribution vehicles is 93.5%.  Figure 13 compares the estimated delivery time of the orders.

As in Figure 13, 15 orders can be delivered within a given distribution time, effectively reducing the distribution penalty cost caused by early arrival or delay after CO. The total cost incurred by the initial scheduling optimization through the collaboration of P-D logistics linkage is expected to be 29,189 RMB. Specifically, the production cost is 23,231 RMB, the storage cost is 4,103 RMB, the distribution cost is 1,855 RMB, and the penalty cost is 0 RMB. Then, the optimization result is modified. The modified dynamic vehicle scheduling result is counted in Figure 14. The modified path numbers are: A1: [0–2 (14) - 9 (10) - 16 (15) - 7 (17) - 0], B1: [0–13 (14) - 5 (16) - 12 (15) - 3 (14) - 0], C1: [0–4 (12) - 11 (13) - 1 (11) - 8 (11) - 0], and D1: [0–10 (18) - 6 (14) - 15 (13) - 14 (13) - 0].  Figure 15 analyzes the dynamically optimized delivery time of orders.

As in Figure 14, after the new dynamic demand is added, the distribution of all orders can be completed by using four distribution vehicles. The load rates are 86%, 91%, 94%, and 89%, respectively, and the average load rate is 90%. As in Figure 15, with the interference of dynamic demand, all orders can also be delivered within a given distribution time, eliminating the adverse impact of dynamics.

P-D's dynamic modification and optimization results corroborate that the random emergence of dynamic demand changes the scheduling plan made in advance by the two subsystems of P-D. However, due to the timely and effective online collaborative operation and independent linkage DM of P-D, each DM unit dynamically adjusts its operation state according to the dynamic interference. The adverse effects caused by dynamic interference are effectively eliminated. The results are detailed in Figure 16:

As in Figure 16, the proposed P-D logistics linkage method to dynamically modify the initial planning results has significant advantages in reducing various costs than nonlinkage. After linkage correction, the production, storage, distribution, penalty, and total system costs are lower than those without linkage.

### 4.2. Sensitivity Analysis

Based on the initial planning, the present work analyzes the impact of linkage DM and nonlinkage DM on P-D operation with different interference degrees. The effectiveness of DM linkage is verified in dealing with active interference. As a result, changes of five indexes are summarized, including production cost, storage cost, penalty cost, distribution cost, and total system cost. The effects of linkage and nonlinkage DM with different periods and requests are compared and analyzed. Sensitivity analysis is conducted under other requests.  Figure 17 reflects the cost changes under different requests.

From Figure 17, with the steady increase of new demands, the production, storage, penalty, distribution, and total system costs rise. Presumably, the increasing demand claims more production and distribution resources, resulting in the upsurging resource utilization cost. Given a few new orders, the difference of various costs under linkage operation and nonlinkage operation is not obvious. The small amount of new demand has probably not exceeded the resource capacity of the production and operation system. Therefore, the new demand can be met in time even without linkage. By comparison, when new demands continue to climb up, linkage operation will show significant advantages in reducing costs than nonlinkage operation. Possibly, there is a threshold for the number of new demands. Once the threshold is reached, the production department under nonlinkage operation can no longer meet the demand timely with its in-department resources. At this time, through linkage operation, external resources are introduced to make up for the lack of resources and complete the production of new demand on time. Without linkage, the demand will not be completed on time. The order queueing time will increase greatly in the warehouse, resulting in a significant increase in storage and penalty costs.

Management enlightenment: When the quantity of new demand changes, the cost of linkage operation is lower than that of nonlinkage operation. When the number of new demands is small, the cost-effectiveness of linkage operation over nonlinkage operation is insignificant. At this time, the production ENTs can selectively adopt linkage operation according to their conditions. As the number of new demands transcends a threshold, the cost-effectiveness of linkage operation is significantly better than that of the nonlinkage operation. Then, production ENTs should actively adopt linkage operations to respond to dynamic demands.

Furthermore, Figure 18 analyzes the cost changes under different order initiation times.

As in Figure 18, little difference is found between the P-D costs of the linkage and nonlinkage operations for an early order initiation time. Every ENT link is not fully loaded at this stage, so the DM link has a potential optimization room. Thus, the DM link can make internal adjustment in P-D and coordinate the P-D links under an early order initiation. Doing so ensures that the dynamic order can be delivered on time. At this time, the storage cost and penalty cost of linkage operation are smaller than nonlinkage operation. However, not much optimization space will be available when an order is initiated after a specific time point. This will result in a similar impact of linkage operation and nonlinkage on storage and penalty costs. Therefore, an early initiation new order will greatly impact the production system. At this time, the total system cost utilizing linkage operation is significantly lower than nonlinkage operation. However, linkage operation costs are greater than nonlinkage operations given a delayed new order.

Management enlightenment: when dynamic orders appear earlier, the cost of linkage operation is lower than that of nonlinkage operation due to the ample optimization space of the production system. Therefore, for an early initiation order, production ENTs should actively carry out linkage operations as soon as possible. With the postponement of the start-up time of new orders, the space limitation of linkage optimization will also be enhanced. The linkage operation often increases the resource investment, with an insignificant optimization effect, resulting in the overall rise of the total system cost. Therefore, the production ENTs should adopt the nonlinkage method to address delayed dynamic demands.

## 5. Conclusion

The problems of P-D DM logistics linkage in the dynamic production environment are analyzed through global optimization to minimize the impact of active interference in the P-D links. Consequently, a set of solutions is proposed, including the architecture and mechanism of P-D DM logistics linkage. The contributions and conclusions are as follows:

1. Based on DT, the dynamic virtual simulation of P-D logistics linkage is carried out, and the framework and mechanism of P-D DM logistics linkage are constructed.
2. The case study shows that the production cost, storage cost, distribution cost, penalty cost, and total system cost of the optimized linkage are 24,943 RMB, 3,393 RMB, 2,167 RMB, 0 RMB, and 30,503 RMB, respectively. The total cost is 3.7% lower than that of a nonlinkage system. Sensitivity analysis shows that ENT managers should adjust the linkage operation state to reduce the manufacturing cost according to different requests.

## Figures and Tables

**Figure 1:** P-D logistics linkage.

**Figure 2:** Digital twins-enabled P-D linkage DM architecture.

**Figure 3:** Architecture of the operation environment.

**Figure 4:** P-D linkage DM mechanism based on DT.

**Figure 5:** Composition of GA.

**Figure 6:** Operation steps of GA.

**Figure 7:** Crossover demonstration based on GA.

**Figure 8:** Mutation operation based on GA.

**Figure 9:** CO of P-D logistics linkage.

**Figure 10:** Basic information of customers.

**Figure 11:** Basic information of distribution vehicles.

**Figure 12:** Optimization results of vehicle scheduling.

**Figure 13:** Estimated delivery time of the orders.

**Figure 14:** Optimization results of vehicle scheduling.

**Figure 15:** Dynamic optimization of delivery time.

**Figure 16:** Cost information.

**Figure 17:** Cost changes under different requests: (a) production cost, (b) total system cost, (c) storage cost, (d) penalty cost, and (e) distribution cost.

**Figure 18:** Cost changes under different order initiation time: (a) production cost, (b) storage cost, (c) distribution cost, (d) total system cost, and (e) penalty cost.

**Table 1:** Hypotheses.

Number	Hypotheses
1	A product consists of multiple subproducts produced and manufactured in different workshops
2	Each order has the same process, and each machine only processes one order at a particular time
3	The processing is not interrupted, and the machine failure is not considered
4	Warehouse the products in time and all derivatives of the same order shall be ready for delivery
5	The warehouse capacity is large enough to ignore the product handling time (warehousing and loading)
6	The speeds of delivery vehicles are the same, without overload, and the limit on delivery distance
7	Vehicle faults and external factors are not considered
8	The distance between the warehouse and each customer is known, and the distance between customers is known
9	The vehicle returns to the factory after completing the task

**Table 2:** Parameter symbols.

Symbols	Description
*P*	Number of production workshops
*N*	Number of the orders to be processed
*D*_*i*_	The delivery date of order *i*
*Q*_*i*_	Product quantity of order *i*
*j*	Production process
*Mj*	Number of optional equipment for operation *j*
*P*	Workshop number, *p* = 1, 2,…, *p*
*i*	Order no.
*α*_*T*_	Number of new orders at time *T*
*Q*_*i*_^*p*^	Product quantity of order *i* in workshop *p*
*j*	Operation no
FC_pro_^*p*^	The fixed production cost of workshop *p*
*T*_*ijk*_*j*__^*p*^	Unit processing time of operation *j* of order *i* on machine *k*_*j*_ in workshop *p*
*k*_*j*_	Number of processing equipment of operation *j*
VC_pro_^*p*^	The variable production cost of workshop P
*t*_off,*i*_^*p*^	Completing time of order *i* in workshop *p*
*x*_*ijk*_*j*__	Production decision variable, the *j-*th operation of order *i* on equipment *k*_*j*_
MT_*i*_^*p*^	Processing time of order *i* on processing equipment in workshop *p*
*K*	Vehicle no.
FC_dis_^*k*^	Fixed cost of vehicle *k*
*z*_*ak*_	Distribution decision variable, whether the products of customer *a* are distributed by vehicle *k*
*S*_*a*_	Customer *a*'s service time
*t*_*e*_*ij*__^*P*^	Finishing time of process *j* of order *i* in workshop *P*. Ending time
*t*_*in*,*i*_^*p*^	Warehousing time of order *i* in workshop *P*
*t*_war,*i*_^*p*^	Storage time of order *i* in the production workshop *p*. Storage time
*C*	Number of customers
*V*	Customer and warehouse collection
*E*_*Tc*_	Earliest delivery time allowed by customer *c*
*K*	Vehicle assembly
*m*	Number of vehicles used
*Q*_*k*_	Maximum loading capacity of vehicle *k*
VC_war_	Unit storage cost
*y*_*abk*_	Distribution decision variables
*t*_*ab*_	Travel time from customer *a* to customer *b*
*Q*_*c*_	Customer *c*'s delivery volume
*λ*	Penalty coefficient for vehicles not arriving at the delivery section
*t*_*s*_*ij*__^*p*^	Processing of operation *j* on order *i* in workshop *p*. Producing time
*t*_out,*i*_^*p*^	Delivery time of order *i* in workshop *p*
*C*	Number of customers
LT_*c*_	Latest delivery time allowed by customer c
*Tc*	Delivery time of customer *c*
VC_dis_^*k*^	Unit distribution cost of vehicle *k*
*d*_*ab*_	Distance from customer *a* to customer *b*

**Table 3:** Some information of ENT H.

Order no.	Production quantity			Total orders	Delivery date	Latest delivery date
	Workshop 1	Workshop 2	Workshop 3			
1	4	3	3	11	12:00	14:00
2	5	7	4	12	10:30	11:30
3	3	3	2	24	12:00	14:00
4	4	3	5	15	11:00	12:00
5	4	9	1	16	11:00	12:00
6	3	7	6	17	12:00	13:00
7	7	4	7	14	11:00	12:00
8	3	3	8	11	12:00	14:00
9	3	7	3	10	10:00	12:00
10	9	3	4	18	12:00	14:00
11	7	3	5	13	11:30	12:30
12	5	9	6	15	11:30	12:30
13	4	7	2	14	11:00	14:00
14	6	4	3	16	12:00	14:00
15	4	5	4	17	12:00	14:00

## Data Availability

The data used to support the findings of this study are included within the article.
